# *Cornu aspersum* mucin attenuates indomethacins-induced gastric ulcers in mice via alleviating oxidative stress and inflammation

**DOI:** 10.1016/j.heliyon.2023.e15677

**Published:** 2023-04-22

**Authors:** Maha B. Salem, Mohamed Elzallat, Dina Mostafa Mohammed, Safia Samir, Olfat A. Hammam, Marwa Tamim A. Abdel-Wareth

**Affiliations:** a Pharmacology Department, Theodor Bilharz Research Institute, Giza, Egypt; b Immunology Department, Theodor Bilharz Research Institute, Giza, Egypt; c Nutrition and Food Sciences Department, National Research Centre, Giza, Egypt; d Biochemistry and Molecular Biology Department, Theodor Bilharz Research Institute, Giza, Egypt; e Pathology Department, Theodor Bilharz Research Institute, Giza, Egypt; f Environmental Research Department, Theodor Bilharz Research Institute, Giza, Egypt

**Keywords:** Gastric ulcer, Indomethacin, *Cornu aspersum*, Mucin, Oxidative stress, Inflammatory markers

## Abstract

In the past three decades, a significant progress has been made in the prevention and treatment of gastric ulcers. The incidence of the disease has decreased, but gastric ulcer is still a medical problem. Currently, the available drugs for gastric ulcer treatment have many side effects; therefore, searching for new and safe therapeutic agents is mandatory. The present study aims to investigate the gastroprotective potential of *Cornu aspersum* (*C. aspersum*) mucin against gastric ulcers, and the mechanisms related to oxidative stress and inflammation. *C. aspersum* mucin was collected from 50 snails. The characteristics of *C. aspersum* mucin (chemical and microbiological) were evaluated. Mice were pretreated with famotidine and *C. aspersum* mucin (7.5 and 15 ml/kg b.w.) for 5 days, and then gastric ulcers were induced by indomethacin. Macroscopic examination, biochemical estimations, and Quantitative real-time PCR were carried out. Also, histopathological and immunohistopathological examinations were evaluated. We found that the high dose of the mucin significantly decreased the gastric mucosal malondialdehyde (MDA) and nitric oxide (NO) contents as well as interleukin 1β (IL-1β) and nuclear factor kappa β (NF-ҡB) expression, and inducible nitric oxide synthase (iNOS) immunostaining. It also increased the gastric mucosal GSH and catalase contents as well as hemoxygenase-1 (HO-1) and nuclear factor-erythroid 2-related factor 2 (Nrf2) expressions with regressions in gastric mucosal lesions. In conclusion, *C. aspersum* mucin could be a potential therapeutic candidate to protect against gastric ulceration.

## 1 Introduction

Peptic ulcer disease (PUD) represents a common gastroenterological disorder, affecting 4 million people each year worldwide, with complications reported in 10–20% of patients [1]. The annual incidence of PUD ranges between 0.10% and 0.19%, with a significant reduction in the last decades due to several therapeutic improvements in the prevention and treatment such as the use of proton pump inhibitors (PPI) and eradication therapy for *Helicobacter pylori* (*H. pylori*) [2]. Unfortunately, PUD is frequently associated with severe complications, including heavy bleeding, perforation, gastrointestinal obstruction, and malignancy [3].

*H. pylori* was discovered in 1983 by Barry J. Marshall and Robin Warren [4]. They deciphered its role in gastritis and peptic ulcer disease and have been awarded that year's Nobel Prize in Physiology and Medicine [5]. It is widely accepted that *H*. *pylori* infection is followed by the induction of inflammatory changes in gastric mucosa that may persist for decades without causing any gastric disturbances. However, in a small percentage of adult patients it may initiate chronic atrophic inflammatory changes of the stomach corpus and associated with an increase in gastrin expression. This disturbance increases the number parietal cells and their acid secretion leading to an increase in acid load damages that resulting in ulcers formation. Furthermore, mucosal cells can be transformed into malignant cells [6]. Moreover, *H. pylori* infection is associated with several extra-gastric pathologies in the digestive system, such as extra-gastric mucosa-associated lymphoid tissue-lymphoma [7], gallstones [8], non-alcoholic fatty liver disease [9], hepatocellular carcinoma [10], and acute pancreatitis [11].

Indomethacin (IND) is non-steroidal *anti-inflammatory* drug that inhibits cyclo-oxygenase-1 in the gastrointestinal tract leading to a reduction of prostaglandin secretion and its cytoprotective effects in gastric mucosa. This causes an increment in pepsin activity and acid production beside a decrease in mucus and bicarbonate secretion which leads to higher the susceptibility to mucosal injury [12]. Additionally, IND promotes lipid peroxidation and reactive oxygen species (ROS) generation in the stomach mucosa [13]. Consequently, IND can be used to induce gastric ulcers in an experimental model [14].

Several pathways, including oxidative stress and inflammation, are involved in gastric ulcer pathogenesis and progression [15,16]. Moreover, ROS accumulation oxidizes proteins and lipids, leading to enhancing the gut permeability, stimulating macrophages, activating the nuclear factor kappa β (NF-ҡB) signaling pathway, and releasing proinflammatory cytokines like interleukin 1β (IL-1β), which worsen the gastric ulcer [17]. Nitric oxide synthase (NOS) is another critical player in this process and is responsible for the production of endogenous nitric oxide (NO) [18]. On the other hand, nuclear factor-erythroid 2-related factor 2 (Nrf2) and hemoxygenase-1 (HO-1) are critical for gastroinstestinal protection because they are responsible for the restoration of the antioxidant defense [19]. Moreover, Nrf2 has been shown to suppress NF-κB, thus inhibiting the signaling of proinflammatory cytokines which play a role in protecting stomach against ulcers induced by IND or other insults [18].

*Cornu aspersum* (*C. aspersum*) belongs to phylum Mollusca, class Gastropoda, order *Stylommatophora*, family *Helicidae* [20]. *Cornu aspersum* was classified under the name *Helix aspersa* for over two centuries, but the prevailing classification now places it in the genus *Cornu*. Generally, *C. aspersum* produces mucin as a dense secretion that covers the external surface of the snail by salivary epidermal glands when the snail injured or heavily irritated, and has many functions in the life of the snail as it possesses adhesive, emollient, protective, and reparative properties [21]. Recently, *C. aspersum* mucin has been used to treat different diseases such as skin and lung diseases like asthma, pneumonia, and pulmonary phthisis [22,23]. Additionally, *C. aspersum* mucin exhibits significant biological features such as antibacterial activity and wound healing ability [24] due to mucin contains essential components such as elastin, collagen, glycolic acid, and allantoin, which play a key role in minimizing the damage triggered by inflammation and oxidative stress [22,25,26].

Searching for new safe drugs of natural origin to treat stomach ulcers is much urgently. Consequently, this study was performed to evaluate the protective effects of the extracted mucin from *C. aspersum* in experimental gastric ulcers induced by IND.

## 2 Materials and methods

### 2.1 Mucin collection

*C. aspersum* snails were collected from different locations in Giza Governorate and transferred to the laboratory, where they were put in plastic cages containing sterilized mud on their bottoms [27]. These cages had special covers that were tightly placed and allowed snails to breathe. The snails were kept under laboratory conditions, sprayed with water, and fed fresh lettuce leaves for one week, but deprived from food three days before mucin extraction [26].

Each individual snail was washed thoroughly with distilled water to remove dirt and feces, and then its pedal glands in the foot region were manually poked with a sterile cotton swab tip to stimulate mucin secretion [23]. Finally, the harvested mucin was put in a sterile falcon tube and kept at −80 until being used.

About 120 ml of crude mucin was collected from 100 snails (2 kg). Before analyzing and using the harvested mucin, it was firstly filtered using a coarse filter, and then serially filtered using three different filters of lower pore sizes (10 μm-1 μm–0.22 μm) and finally stored at 4 °C.

### 2.2 *Chemical characterization of C. aspersum* mucin

*C. aspersum* mucin was analyzed for its physical properties according to Ref. [28]. The glycolic acid and allantoin contents were chemically analyzed using Shimadzu high-performance liquid chromatography (HPLC) (CLASS-M10A, Tokyo, Japan) [29]. Qubit Protein Assay Kit (Thermo, USA) was used to measure total protein concentration. Elastin and collagen were determined by Fastin Elastin assay and Sircol Collagen assay, respectively [30,31]. All-trans-retinol, and 13-cis-retinol, besides vitamins E and A, were measured according to Ref. [32], while vitamin C was determined spectrophotometrically according to Ref. [33]. Vitamins B1 and B2 were detected by the acid hydrolysis method according to Ref. [34], whereas vitamins B3, B6, and B12 were detected according to Ref. [35]. At the same time, the minerals in *C. aspersum* mucin were measured by atomic absorption spectroscopy [36].

### 2.3 Microbiological characterization

In order to exclude any microbial contamination, 100 μl of *C. aspersum* mucin was cultured onto Tryptic Soy agar (TSA) plates (Biomerieux, Italy), and the number of colony-forming units (CFU) was observed after incubation for 24 and 48 h at 37^°^Cto determine whether there was bacterial contamination [36]. The bacterial contamination was identified by Gram staining (Liofilchem, Italy). Regarding fungal contamination, it was evaluated by inoculating Sabouraud dextrose agar (SDA) plates (Biomerieux, Italy) with 100 μl of *C. aspersum* mucin, and observing fungal growth after 3–7 days of incubation at 28 °C.

### 2.4 Experimental animals

Male Swiss mice, weighing 20–30 g, were purchased from the animal house unit, Theodor Bilharz Research Institute (TBRI), Giza, Egypt. Mice were housed in standard conditions of temperature (25 ± 2 °C), light cycle (12-h light/dark cycles), and humidity (50 ± 15%) with free access to water and food. The study was approved by TBRI Institutional Review Board (IRB) {PT: 664; FWA 0010609; issue date (1/2022) and expiry date (1/2023)}in accordance with the United Kingdom's Animals (Scientific Procedures) Act, 1986 and associated guidelines, EU Directive 2010/63/EU for animal experiments (Publication No. 85-23, revised 1985).

### 2.5 Drugs

The drugs used in this study were IND (Indocin®, Kahira Pharm. & Chem. Ind. CO., Cairo, Egypt, batch number: 2120001) and famotidine (FAM) (Famotin®, Memphis Pharm. & Chem. Ind. CO., Giza, Egypt, batch number: 321026).

### 2.6 IND-induced acute gastric ulcer

IND-induced acute gastric ulcer was carried out according to Ref. [37]. Briefly, the mice were refrained from eating food for 24 h before receiving a single oral dose of IND (18 mg/kg) on the 5th day of the study period.

### 2.7 Experimental design

Forty eight mice were randomly allocated into 8 groups (6 mice each). Group 1 (normal control): mice received distilled water (15 ml/kg) and treated with IND vehicle (2% Cremophore-El; Sigma-Aldrich, St. Louis, MO, USA) at the last day of the study. Groups 2–4: normal mice were orally administered with FAM (40 mg/kg b.w.), a low dose of *C. aspersum* mucin (7.5 ml/kg b.w.), and a high dose of *C. aspersum* mucin (15 ml/kg b.w.), respectively for 5 *consecutive* daysand treated with IND vehicle at the last day of the study. Group 5 (ulcerated control): mice were given a single oral dose of IND in the form of aqueous suspension in 2% Cremophore-El on the 5th day of the study period. Groups 6–8: mice were orally administered respectively with FAM (40 mg/kg b.w.) in the form of aqueous suspension in 2% Cremophore-EL [38], a low dose of *C. aspersum* mucin (7.5 ml/kg b.w.), and a high dose of*C. Aspersum* mucin (15 ml/kg b.w.) [23]. All the treatments were administered once daily for 5 *consecutive* days and the last dose was 2 h prior to IND administration. *Four hours later, the mice were euthanized under light anaesthesia, and the stomach was surgically removed and washed with* phosphate saline buffer*. Then, the stomach was opened along its greater curvature for macroscopical examination.* Immediately after ulcer scoring, the stomach was divided into 3 parts; the 1st part was used for RNA extraction. The 2nd part was homogenized before being used to ensure the maximal release of the oxidative stress enzymes from the tissue, whereas, the last part was formalin-fixed for histological and immune-histochemical assessment.

### 2.8 Macroscopic examinations

Ulcer scoring in the IND-treated mice was determined using the procedures described by Ref. [39]. Briefly, stomach lesion width (mm) and length (mm) were determined using a Vernier caliper. Then, the mean ulcer score/group was expressed as ulcer index U.I. and calculated as follows:

(1) U.I.=[Ulceratedarea/totalstomacharea]×100

Finally, the gastric mucosal lesions were evaluated and scored as shown in Table 1.

**Table 1:** Scores for the mucosal lesions.

Macroscopic appearance	Score
No ulcer	0
1–5 petechiae (<1 mm)	1
6–10 petechiae (<1 mm)	2
>10 petechiae (<1 mm)	3
Small linear ulcer (<2 mm)	2
Medium linear ulcer (2–4 mm)	3
Large linear ulcer (>4 mm)	4

### 2.9 Biochemical estimations

To detect the oxidative and antioxidant cascades, reduced glutathione (GSH) [40], catalase [41], malondialdehyde (MDA) [42], and NO [43] were measured by commercial kits (Biodiagnostic Company, Egypt).

### 2.10 Quantitative real-time PCR

Total RNA was extracted from stomach tissues using RNeasy Mini kit (Qiagen, USA). Quanti Tect Reverse Transcription Kit (Qiagen, USA) was used to reverse-transcribe total RNA to cDNA. The PCR reactions were performed using SYBR Green PCR Mastermix kit (Qiagen, USA). The thermal cycling conditions were: 3 min at 95 °C, 40 cycles at 95 °C for 10 s, 55 ^°^C step for 30 s, and a 72 °C step for 30 s. Relative expression of the target genes was calculated against the reference gene, β-actin. The sequences of primer were shown in Table 2 [44].

**Table 2:** The primmer sequence and annealing temperatures for quantitative real-time PCR.

Target gene (s)	Amplicon length (bp)	Primer sequence
Nrf2	225	Forward primer: 5′-ATGATGGACTTGGAGCTGCC-3′
		Reverse primer: 5′-TTGTAACTGAGCGAAAAAGGCTTT-3′
HO-1	127	Forward primer: 5′-TTCAGAAGGGCCAGGTGACC-3′
		Reverse primer: 5′-AAGTAGACAGGGGCGAAGACTGG-3′
NF-ҡB	78	Forward primer: 5′-CTGGTGGACACATACAGGAAGAC-3′
		Reverse primer: 5′-ATAGGCACTGTCTTCTTTCACCTC-3′
IL-1β	72	Forward primer: 5′-GCTGCTACTCATTCACTGGCAA-3′
		Reverse primer: 5′-TGCTGCTGGTGATTCTCTTGTA-3′
Beta actin	118	Forward primer: 5′-GGGAATGGGTCAGAAGGACT-3′ Reverse primer: 5′-CTTCTCCATGTCGTCCCAGT-3′

### 2.11 Histopathological and immune-histopathological examinations

Parts of the stomach tissues from each group were immediately formalin-fixed for 24 h. Specimens were sliced and stained with hematoxylin-eosin (H & E) and toluidine blue stain and then examined under a light microscope. Immunoperoxidase staining of stomach tissues was done using monoclonal antibodies against *inducible nitric oxide synthase* (iNOS) [45] and examined by a light microscope.

### 2.12 Statistical analysis

Data were expressed as mean ± SE. A one-way ANOVA test followed by Tukey post-*hoc* test was used to evaluate the significant differences between the mean values of studied groups using SPSS software, version 22.0 (Chicago, IL, USA). *p* < 0.05 was considered statistically significant [46].

## 3 Results and discussion

Gastric ulcers encompass a diverse group of diseases characterized by mucosal lesions and inflammation with multifactorial and complex etiologies [47]. Inflammation, oxidative stress, and neutrophil infiltration have all been involved in the pathophysiology of gastric ulcers [48].

The usual approaches in gastric ulcers treatment are based on histamine type 2 receptor blockers and PPIs. Unfortunately, these classes of drugs may lead to serious side effects when used for a long time [49]. Therefore, using therapeutic agents with potent antioxidant and anti-inflammatory activities is supposed to be an effective strategy for gastric ulcers prevention.

Snail mucin has recently been shown to be able to treat and protect against a number of illnesses because of its antioxidant and anti-inflammatory properties [36,50]. This mucin is a dense and viscid secretion that coats the snail's external surface and is produced by salivary epidermal glands. It has many functions during the life of snails as it possesses emollient, adhesive, reparative, and protective proprieties [21].

This study provided a deep understanding of the mechanistic effects of *C. aspersum* mucin in protecting against IND-induced gastric ulcers in mice, taking into consideration Nrf2/Ho-1 pathway and determining the crucial role of iNOS/NO.

### 3.1 Chemical and microbiological characterization of C. aspersum mucin

Characterization of the biological properties of *C. aspersum* mucin requires standardization of the purification procedures as well as chemical and microbiological analyses of the extract. In the present study, the chemical composition of *C. aspersum* mucin results in Table 3 indicated that *C. aspersum* mucin had unique features, as it has high glycolic acid (210 ± 3.82 mg/L) and collagen contents (85 ± 0.65 mg/L) in addition to allantoin (20 ± 1.9 mg/L) and elastin (0.099 ± 0.0005 g/100 g). Moreover, the microbial characterization revealed that *C. aspersum* mucin was sterile as no bacteria or fungi were observed. These results were in line with [25], who reported that many of these components, including glycolic acid, allantoin, collagen, and elastin, play important roles in gastric mucosa protection and homeostasis. Furthermore [51], demonstrated that there were many compounds found in snail slime that contribute to its particular protective activity, such as copper, which has been shown to have anti-ulcer properties.

**Table 3:** Qualitative and quantitative chemical and microbiological analysis of *Cornu aspersum* mucin.

Specification	Specification value (Mean ± SE)
Aspect	Clear fluid
Color	Light amber
Smell	Odorless
Ph	4.80 ± 0.10
Density	1.04 ± 0.01
Dry residual (g/ml)	3 ± 1.53
Yield (%)	0.17
Proteins (mg/L)	250 ± 2.52
Glycolic acid (mg/L)	210 ± 3.82
Allantoin (mg/L)	20 ± 1.9
Polyphenols (mg/L)	80 ± 1.51
Elastin (g/100 g)	0.099 ± 0.0005
Sugars (g/L)	0.029 ± 0.01
Collagen (mg/L)	85 ± 0.65
Gram + (CFU)	0
Gram – (CFU)	0
Fungi (CFU)	0
All-trans-retinol (μg/100 g)	10 ± 0.58
13-cis-retinol (μg/100 g)	9 ± 1.15

Regarding vitamin content, our results in Table 4 revealed that 100 g of mucin contained high concentration of vitamin B6 (19.11 ± 0.11 μg/ml), followed by vitamins B3 (9 ± 1.53 μg/100g) and B12 (9 ± 0.2 μg/100g), besides a considerable content of vitamin B1 (3.15 ± 0.005 μg/ml), vitamins A (0.99 ± 0.01 μg/ml), B2 (0.75 ± 0.22 μg/ml), C (0.15 ± 0.006 mg/kg) and E (0.11 ± 0.003 mg/kg).This vitamin content gave mucin more value as [52] demonstrated that vitamins have critical roles in human digestion, metabolism, and immunity.

**Table 4:** Vitamin contents of *Cornu aspersum* mucin.

Vitamin	Concentration (Mean ± SE)
E (mg/kg)	0.11 ± 0.003
C (mg/kg)	0.15 ± 0.006
A (μg/ml)	0.99 ± 0.01
B1 (μg/ml)	3.15 ± 0.005
B2 (μg/ml)	0.75 ± 0.22
B3 (μg/100 g)	9 ± 1.53
B6 (μg/ml)	19.11 ± 0.11
B12 (μg/100 g)	9 ± 0.2

The particular protective action of *C. aspersum* mucin may be due to its mineral components (Table 5). The highest mineral concentration was that of calcium (1350 ± 3.05 mg/kg) followed by potassium (1065 ± 2.88 mg/kg), phosphorus (955 ± 1.01 mg/kg) and sodium (932 ± 2.52 mg/kg), In addition to magnesium (175 ± 2.52 mg/kg) and iron (6.01 ± 0.03 mg/kg). Also, *C. aspersum* mucin contained trace elements such as Cr (0.009 ± 0.0005 mg/kg), Cu (5.09 ± 0.1 mg/kg), Hg (0.25 ± 0.01 μg/kg), Cd (0.019 ± 0.001 μg/kg), Co (0.001 ± 0.0006 μg/kg), Ni (0.95 ± 0.04 μg/kg), Zn (1.35 ± 0.02 mg/ml) and Mn (0.69 ± 0.01 mg/ml).

**Table 5:** Minerals and trace elements contents of *Cornu aspersum* mucin.

Minerals and Trace Elements	Concentration (Mean ± SE)
Ca (mg/kg)	1350 ± 3.05
Mg (mg/kg)	175 ± 2.52
Fe (mg/kg)	6.01 ± 0.03
Na (mg/kg)	932 **±** 2.52
P (mg/kg)	955 ± 1.01
K (mg/kg)	1065 ± 2.88
Cr (mg/kg)	0.009 ± 0.0005
Cu (mg/kg)	5.09 ± 0.1
Hg (μg/kg)	0.25 ± 0.01
Cd (μg/kg)	0.019 ± 0.001
Co (μg/kg)	0.001 ± 0.0006
Ni (μg/kg)	0.95 ± 0.04
Zn (mg/mL)	1.35 ± 0.02
Mn (mg/mL)	0.69 ± 0.01

### 3.2 Macroscopic examinations

The stomach of normal controls showed no signs of ulceration or hemorrhagic lesions (Fig. 1A). Moreover, the stomach of normal mice received FAM, low dose of *C. aspersum* mucin or high dose of *C. aspersum* mucin showed no signs of ulceration or hemorrhagic lesions (Fig. 1A). In contrast, the stomach of ulcerated controls showed visible hemorrhagic lesions and severe ulcers (Fig. 1A). Compared with the normal controls, the U.I. of the ulcerated controls was increased to 7.45 mm^2^withan ulcer score of 2.83 (Fig. 1B and C). Pretreatment with FAM reduced hemorrhagic lesions and ulceration (Fig. 1A) and caused a 67.60% ulcer protection effect with U.I. of 2.35 mm^2^ (Fig. 1C). Similarly, pretreatment with *C. aspersum* mucin at a low dose and high dose (Fig. 1A) significantly improved hemorrhagic lesions or ulceration, and significantly decreased (p < 0.05) the U.I. to 3.53 and 1.76 mm^2^, respectively compared with the ulcerated controls (Fig. 1C). Moreover, pretreatment with *C. aspersum* mucin at a high dose (15 ml/kg) provided a more pronounced effect in ulcer score (Fig. 1B). These results demonstrated that *C. aspersum* mucin offered a considerable protection against gastric ulcers caused by IND.

**Fig. 1:** Macroscopic inspection of the mice gastric mucosa (A), effect of *Cornu aspersum* mucin on gastric ulcer score (B) and gastric ulcer index (C).Black arrows indicate ulcer. Values were presented as means of 6 mice ± SE.^b, c, d^ significantly different (*p* < 0.05) from Indomethacin (IND), Famotidine (FAM), and low dose of *C. aspersum* mucin groups, respectively.

### 3.3 Biochemical estimations

ROS generated in gastric tissues by activated neutrophils was associated with delayed stomach ulcer healing [53]. Intracellular antioxidants such as catalase and GSH could neutralize the generated ROS [54].

In normal mice received FAM, low dose of *C. aspersum* mucin or high dose of *C. aspersum* mucin, the stomach tissue contents of MDA, GSH, catalase, and NO showed no significant difference when compared with normal control group. The stomach tissue contents of MDA, GSH, catalase, and NO were indicated in Fig. 2A–D. In the ulcerated controls, gastric lipid peroxidation expressed as MDA and NO were significantly increased (*p* < 0.05) by 2.88 and 3.46-folds, along with significant depletion (*p* < 0.05) in the contents of the antioxidant enzymes; GSH, and catalase by 2.29 and 2.46-folds, respectively in comparison with normal controls.

**Fig. 2:** Effect of *Cornu aspersum* mucin on gastric mucosa (A) malondialdehyde (MDA), (B) reduced glutathione (GSH), (C) catalase, and (D) nitric oxide (NO) contents in mice. Values were presented as means of 6 mice ± SE.^a, b, c, d^ significantly different (*p* < 0.05) from normal, Indomethacin (IND), Famotidine (FAM) or low dose of *C. aspersum* mucin groups, respectively.

Pretreatment with FAM or *C. aspersum* mucin, at a high dose, normalized gastric MDA contents. Our results were in harmony with [55] who stated that IND intoxication resulted in a significant increase in the level of MDA, and a significant decrease in the activities of GSH, and catalase. Yet, pretreatment with *C. aspersum* mucin at a low dose significantly reduced (p < 0.05) the level of MDA by 26.52% compared with the ulcerated controls. While The depleted GSH and catalase contents were significantly replenished (*p* < 0.05) by pretreatment with FAM by 91.39% and 77.90%, respectively, *C. aspersum* mucin at a low dose by 38.56% and 67.68%, respectively, and *C. aspersum* mucin at a high dose by 88.56% and 116.57%, respectively when compared with the ulcerated controls. Moreover, pretreatment with a high dose of *C. aspersum* mucin normalized gastric NO level. Pretreatment with either FAM or *C. aspersum* mucin, at a low dose, significantly reduced (*p* < 0.05) gastric NO level by 44.04% and 37.50%, respectively, when compared with the ulcerated controls. These findings highlighted the beneficial role of *C. aspersum* mucin in ameliorating oxidative stress resulted from the pathogenesis of gastric ulcer and improving antioxidant capacity.

### 3.4 Effect of C. aspersum mucin pretreatment on the expression of gastric mucosal Nrf2 and HO-1

The Nrf2/HO-1 signaling pathway is crucial for protecting the cells from oxidative stress-induced damage by restoring the antioxidant defenses (Catalase, GSH, and HO-1) [56]. Nrf2 interacts with the negative regulator Keap1 and becomes inactive in the cytoplasm. Oxidative stress leads to dissociation of Nrf2 from Keap1and promotes its translocation from the cytoplasm to the nucleus. This leads to the activation of Phase II enzymes [57]. HO-1 is linked to cyto-protection against oxidative stress and injuries caused by ROS [58].

In normal mice received FAM, low dose of *C. aspersum* mucin or high dose of *C. aspersum* mucin, the relative expressions of the Nrf2 and HO-1 genes showed no significant difference when compared with normal control group. Moreover, the relative expressions of the Nrf2 and HO-1 genes were significantly diminished (p < 0.05) in the ulcerated controls by 2.71 and 1.89-folds, respectively, compared with the normal controls. Our results were in agreement with [58] who stated that the relative expression of Nrf2 gene was reduced in ulcerated group induced by ethanol in type II diabetic rats. Meanwhile, pretreatment with FAM, a low dose of *C. aspersum* mucin*,* and a high dose of *C. aspersum* mucin caused a significant up-regulation of the relative expression of Nrf2 and HO-1 when compared to the ulcerated controls. These results aligned with [59,60], who declared that natural products could modulate the Nrf2/HO-1 pathway and hence restore the antioxidant defense system. This could explain the gastroprotective effects of the *C. aspersum* mucin observed in the pretreated groups (Fig. 3A and B).

**Fig. 3:** Effect of *Cornu aspersum* mucin on gastric mucosa (A) Nuclear factor erythroid 2-related factor 2 (Nrf2), and (B) Hemoxygenase-1 (HO-1) expressions in mice. Values were presented as means of 6 mice ± SE.^a, b, c, d^ significantly different (*p* < 0.05) from normal, Indomethacin (IND), Famotidine (FAM), or low dose of *C. aspersum* mucin groups, respectively.

### 3.5 Effect of C. aspersum mucin pretreatment on the expression of gastric mucosal inflammatory markers

The NF-ҡB transcription regulator, which is responsible for DNA interaction, dimerization, and binding with inhibitory proteins, is known to modulate the oxidative stress, and inflammatory response [61].

As illustrated in Fig. 4A, B), the relative expressions of the gastric inflammatory markers; NF-ҡB and IL-1β. Normal mice received FAM, low dose of *C. aspersum* mucin or high dose of *C. aspersum* mucin showed no significant difference when compared with normal control group. Moreover, the relative expressions of the gastric NF-ҡB and IL-1βwere significantly enhanced in the ulcerated controls by 2.49 and 3.27-folds, respectively compared with the normal controls. Conversely, administration of FAM, a low dose of *C. aspersum* mucin*,* and a high dose of *C. aspersum* mucin significantly reduced (p < 0.05) the relative expression of NF-ҡB by 42.06%, 28.17%, and 36.90% and IL-1β by 36.06%, 30.61%, and 40.00%, respectively when compared with the ulcerated controls. Yet, the superior effect on the reduction of the relative expressions of NF-ҡB and IL-1β was provided by the high dose of *C. aspersum* mucin. The reduction in the relative expressions of NF-κB and IL-1β in *C. aspersum* mucin and FAM pre-treated mice may be due to the ROS scavenging activity of *C. aspersum* mucin and FAM. A previous report had shown that antioxidants can suppress the NF-ҡB activation stimulated by ROS and block the transcription of proinflammatory cytokines such as IL-1β in ethanol-induced gastric ulcers [62].

**Fig. 4:** Effect of *Cornu aspersum* mucin on gastric mucosa (A) nuclear factor kappa-β (NF-ҡB), and (B) Interleukin-1β (IL-1β) expressions in mice. Values were presented as means of 6 mice ± SE. ^a, b, c^ significantly different (*p* < 0.05) from normal, Indomethacin (IND), or Famotidine (FAM) groups, respectively.

Besides oxidative stress and inflammatory response, NO produced by the endothelial NOS and neuronal NOS isoforms has a role in protecting the gastric mucosa. It causes vasodilation that leads to proper gastric micro-circulation and acceleration of repair [63]. Furthermore, NO is associated with inhibiting both the acid secretion and the action of proinflammatory mediators. It also stimulates mucin secretion in the stomach by increasing cyclic guanosine monophosphate levels [64]. However, NOS isoforms induced by proinflammatory cytokines such as IL-1β, and interferon γ, produce a tremendous amount of NO. NO is potentially toxic at these levels and contributes to oxidative stress, leukocyte adhesion, and chemotaxis that promote inflammatory cells infiltration and free radicals production. In the current study, ulcerated controls showed an increment of gastric mucosa NO content. However, pretreatment with either low or high doses of *C. aspersum* mucin and FAM showed a significant decrease in toxic level NO. Our results suggest that *C. aspersum* mucin may affect the NO pathway.

### 3.6 Histopathological and immunohistochemical examinations

The histopathological findings further confirmed our results. Normal gastric tissues revealed a normal histological structure of gastric mucosa where the mucosa has no signs of deterioration (Fig. 5A). Also, normal mice received FAM, low dose of *C. aspersum* mucin or high dose of *C. aspersum* mucin showed a normal histological structure of gastric mucosa (Fig. 5B–D). In contrast, gastric tissues of the ulcerated controls exhibited severe mucosal depletion accompanied by extensive lesions, hemorrhages, intense deterioration, and necrosis. Moreover, in addition to depression of gastric pits, submucosal edema, and severe inflammatory cell infiltration were also observed (Fig. 5E). On the other hand, gastric tissues from FAM and a high dose of *C. aspersum* mucin pretreated groups showed a considerable amelioration of the structural alteration by guarding against gastric mucosal loss. The observed cell infiltrates reduction due to the ameliorative effect of high dose of *C. aspersum* mucin was more remarkable than that observed for FAM (Fig. 5F&H). Additionally, gastric tissue from a low dose of *C. aspersum* mucin pretreated group showed a moderate amelioration of the structural alteration with a reduction in inflammatory cells infiltration (Fig. 5G).

**Fig. 5:** Effect of *Cornu aspersum* mucin on stomach histopathological changes. (A) Normal controls, (B) Normal mice received Famotidine (FAM), (C) Normal mice received low dose of *C. aspersum* mucin, (D) Normal mice received high dose of *C. aspersum* mucin, (E) Ulcerated controls, (F) FAM pretreated group, (G) Low dose of *C. aspersum* mucin pretreated group, and (H) High dose of *C. aspersum* mucin pretreated group. Black arrows indicate epithelium appearance and red arrows indicate edema and leucocytes infiltration (H & E, ×100). (For interpretation of the references to colour in this figure legend, the reader is referred to the Web version of this article.)

Concerning toluidine blue stain, normal mice and normal mice received FAM, low dose of *C. aspersum* mucin or high dose of *C. aspersum* mucin showed normal distribution of mucin secreting cells (Fig. 6A–D), While, IND-intoxicated group exhibited a reduction in the number of mucin secreting cells in gastric mucosa (Fig. 6E). On the other hand, mice pretreated with FAM (40 mg/kg) and the low dose of *C. aspersum* mucin (7.5 ml/kg), respectively showed an increase in the number of mucin secreting cells (Fig. 6F and G). Mice pretreated with the high dose of *C. aspersum* mucin (15 ml/kg) showed a marked increase in the number of mucin secreting cells (Fig. 6H).

**Fig. 6:** Histological section of gastric mucosa in (A) Normal controls, (B) Normal mice received Famotidine (FAM), (C) Normal mice received low dose of *Cornu aspersum* (*C. aspersum*) mucin, (D) Normal mice received high dose of *C. aspersum* mucin, (E) Ulcerated controls, (F) FAM pretreated group, (G) Low dose of *C. aspersum* mucin pretreated group, and (H) High dose of *C. aspersum* mucin pretreated group. Black arrows indicate the mucin secreting cells (Toluidine blue stain, ×200). (For interpretation of the references to colour in this figure legend, the reader is referred to the Web version of this article.)

Regarding iNOS immunostaining, normal mice and normal mice received FAM, low dose of *C. aspersum* mucin or high dose of *C. aspersum* mucin showed few numbers of cytoplasmic positively stained cells (Fig. 7A–D). While the ulcerated controls showed marked numbers of cytoplasmic brownish stained cells (55%) (Fig. 7E and I). In contrast, pretreatment with FAM resulted in few numbers of cytoplasmic brownish stained cells (20%) (Fig. 7F and I). On the other hand, pretreatment with a low dose of *C. aspersum* mucin showed moderate numbers of cytoplasmic positively stained cells (27.50%) (Fig. 7G and I), whereas few numbers of cytoplasmic positively stained cells were observed in mice pretreated with a high dose of *C. aspersum* mucin (11%) (Fig. 7H and I).

**Fig. 7:** Effect of *Cornu aspersum* mucin on stomach inducible nitric oxide synthase (iNOS) immunostaining changes. (A) Normal controls, (B) Normal mice received Famotidine (FAM), (C) Normal mice received low dose of *C. aspersum* mucin, (D) Normal mice received high dose of *C. aspersum* mucin, (E) Ulcerated controls, (F) FAM pretreated group, (G) Low dose of *C. aspersum* mucin pretreated group, and (H) High dose of *C. aspersum* mucin pretreated group. Black arrows indicated expression of iNOS (DAB, IHC, iNOS, ×200), and (I) % of iNOS positively stained cells. Values were presented as means of 6 mice ± SE.^a, b, c, d^ significantly different (*p* < 0.05) from normal, Indomethacin (IND), FAM, or low dose of *C. aspersum* mucin groups, respectively.

The gastroprotective effects of *C. aspersum* mucin may be directly related to its ability to restore the antioxidant defense and reduce the gastric inflammation, and indirectly related to the possibility of hydrochloric acid and IND to bind with *C. aspersum* mucin, which may lower the concentration of these compounds in the gastric content. As a consequence, there may be decreased penetration of gastric mucosa by IND and hydrogen ions, as well as decreased absorption of indomethacin by intestinal mucosa.

## 4 Conclusion

*C. aspersum* mucin exhibited significant gastroprotective effects against IND-induced stomach ulcers. These gastroprotective effects could be due to the restoration of the antioxidant defence system via upregulation of gastric mucosalNrf2 andHO-1 expression and downregulation of IL-1β and NF-κB expressions, as well as diminished lipid peroxidation expressed as gastric mucosa MDA content. Besides, it caused an increase in gastric mucosa GSH and catalase content. These gastroprotective effects could be attributed to the unique active constituents of the mucin could stipulate these gastroprotective effects. Therefore, *C. aspersum* mucin can be considered as a potential therapeutic candidate to protect against gastric ulceration*.*

## Author contribution statement

Maha B. Salem, Dina Mostafa Mohammed: Conceived and designed the experiments; Performed the experiments; Analyzed and interpreted the data; Contributed reagents, materials, analysis tools or data; Wrote the paper. Mohamed Elzallat: Conceived and designed the experiments; Performed the experiments; Analyzed and interpreted the data; Wrote the paper. Safia Samir, Olfat A. Hammam, Marwa Tamim A. Abdel-Wareth: Performed the experiments; analyzed and interpreted the data; wrote the paper.

## Data availability statement

Data will be made available on request.

## Declaration of interest's statement

The authors declare no conflict of interest.

## Additional information

Supplementary content related to this article has been published online at [URL].

## Declaration of competing interest

The authors declare that they have no known competing financial interests or personal relationships that could have appeared to influence the work reported in this paper.

## Funding

This research did not receive any specific grant from funding agencies in the public, commercial, or not-for-profit sectors.
